# Application of Cheerleading Referee Information Management System Based on Data Mining

**DOI:** 10.1155/2022/8912627

**Published:** 2022-08-02

**Authors:** Xueqing Yang, Bo Li

**Affiliations:** ^1^College of Physical Education, Xihua University, Chengdu, Sichuan 610039, China; ^2^Department of Physical Education, Civil Aviation Flight University of China, Guanghan, Sichuan 618307, China

## Abstract

In recent years, China has focused on the development of sports and adopted modern, scientific, and standardized management of referees. Global sports events are becoming increasingly fierce. One of the main links is to manage the referee group and ensure the fairness and impartiality of sports competitions. In sports competition, referees implement sports rules, so the quality of referees directly determines whether sports events are fair and just. Cheerleading operation was introduced into China as a new sports event and spread rapidly in major universities and primary and secondary schools. With the increase of the number of cheerleading athletes, the number of referees also continues to increase. Referees' information management has become the main problem. Therefore, this paper uses data mining technology to design and develop cheerleading referee information management system, uses the system to manage the basic information of cheerleading referees, and analyzes the sanction ability and strength of cheerleading referees. This paper first introduces the basic concept and operational process of data mining algorithm, and C4.5 decision tree algorithm, and support vector machine algorithm. Based on this algorithm, a cheerleading referee information management system is established. Then, we analyze the system structure and demand analysis and design the main structure of the system. Finally, the number of cheerleading referees is analyzed. The highest proportion of referees is 29.5%, the number of referees is 3 to 5 times, and the highest proportion of referees with more than 10 times per year is 59.24%. Using this system to analyze the strength of cheerleading referees, the most influential factor is the lack of on-the-spot experience, accounting for 38.83%.

## 1. Introduction

Large datasets are sorted and processed routinely through data mining in order to discover useful patterns and correlations which may be effective in the whole process of the data analysis. These analyses or examinations are utilized to assist an individual in solving a particular business challenge at hand. Enterprises can be enabled to forecast future trends and make better educated and informed business decisions. These are becoming possible due to the extensive qualities of the data mining techniques and technologies which are developed in order to carry out these task in an effective way. These techniques have numerous applications and could be utilized in almost every era of the business especially in those scenarios where evaluation or extensive analysis is needed.

Cheer-up has a strong sense of rhythm, uniqueness, and fitness. It can highlight the energetic and positive spirit of young people, and it has become one of the most favorite sports of colleges and students. Cheer-up is mainly carried out in colleges and universities. It can attract a large number of students to become check-up athletes or referees and build a complete check-up team. At the same time, the integration of physical education content in cheer-up can stimulate students' learning initiative [1].

Chinese cheer-up referees' information management is still kept on paper, which makes it hard to discover and has less content. As a result, it cannot satisfy the involved parties' fundamental demands for the referees' information management. In order to address this issue and increase the effectiveness of information management, a cheer-up referees' information management system is set up using a data mining algorithm, and data mining technology is used to precisely, scientifically, and safely manage the cheer-up referees' information [2].

The main innovations in this research process are as follows. (1) First, briefly introduce the data mining algorithm used by the system, overview the concept and process of data mining, and describe in detail the two commonly used algorithms in data mining, namely, C4.5 decision tree algorithm and logistic regression algorithm [3]. (2) Analyze the functional and data requirements of the actual system of Chinese cheer-up referees, based on which the main structure design of the system is completed, and the information management system of cheer-up referees based on data mining is established.

## 2. Related Work

Nowadays, people's quality of life is improving day by day. The value of cheerleading in fitness, medical treatment, health care, entertainment, and bodybuilding is sought after by people. However, there is less research on the information management of cheerleading referees. Kim et al. pointed out that the most common types of cheerleading are skill cheerleading and dance cheerleading and further subdivided them into street dance, flower ball, free dance, and jazz dance [4]. Jing studied the cheerleading training in Shandong Province and analyzed the coaches' ability, training, and athletes' quality, which restrict the cheerleading training [5]. In order to increase the quantity and quality of cheerleading coaches and support the school curriculum system in establishing a cheerleading club, Qin analyzed the participation of college cheerleading teams, the current situation of cheerleading athletes, and the team of coaches and analyzed the future development trend of cheerleading in combination with the unique culture of different regions [6]. Zhang created an industrialized system by researching American cheering. It supports the tremendous growth of American cheerleading as the core component of the American sports business [7]. Based on the United States' strong cheerleading history, cheerleading competitions, training methods, and management strategies are used to advance development rights and interests. According to the current situation of cheerleading referee management, the main problems of referee management are uneven level, single physique, lack of scientific research ability, etc. corresponding management measures shall be taken to solve those problems [8]. Li studied the development status of Chinese dance referees from the micro and macro-perspectives, constructed the referees' information management database, and introduced the benign mechanism [9]. Meng used director sports simulation training technology in sports event referee to explain the basic simulation principle and implementation process, which is of great value for the referee simulation system [10]. Fan and Liu deeply studied the computer application in school sports management and proposed that computer technology can comprehensively improve the efficiency of sports management [11]. Cheng and Liu deeply analyzed the characteristics of cheerleading projects, used regenerative training in training cheerleading projects, expected this kind of training to be used in the process of cheerleading training, and formulated cheerleading training plan [12]. Guo introduced cheerleading in secondary vocational schools, colleges, and primary schools to strengthen students' physical quality, give full play to the spirit of cheerleading competition, manage the cheerleading project team in a scientific way, and improve the training results of cheerleading athletes [13].

## 3. Overview of Data Mining Algorithms

Initially, a brief but thorough and rigorous review of the data mining approach is presented below but starting with its definition and then describing its steps one by one.

### 3.1. Concept and Process of Data Mining

Data mining is a process of analyzing and finding datasets. Data mining can find the internal rules and relationships of data and predict the future development trend based on the current data [14]. Data mining can be applied to data warehouse, relational database, advanced database system, and transaction database. Its generation mode is efficient, understandable, potentially valuable, and effective. Generally, the information obtained by data mining reflects three characteristics, namely, effectiveness, predictability, and practicability.

Data mining techniques are being updated and enhanced as information technology advances quickly. Data mining aims to uncover hidden laws or patterns in data in order to provide decision makers a solid data foundation. Data mining is a multi-step, repetitive process. Prior to beginning data mining, it is important to define the mining object, acquire the necessary technology and skills, and advance our understanding of the data and company.  Figure 1 illustrates the data mining process, which primarily involves data preparation, data mining, and knowledge representation:

### 3.2. C4.5 Decision Tree Algorithm

C4.5 algorithm is based on M3 decision tree algorithm. The drawbacks of this algorithm are analyzed and improved. After successful improvement, the accuracy of classification is high and the speed of operation is fast. It has become the most popular decision tree algorithm [15]. The information gain essence of attribute *A* is the unconditional direct values of class *C* in dataset *S*. The unconditional direct values of class *C* is divided according to attribute *A*, which is shown below:

(1) $$\begin{array}{c} \text{Gain}\left(S,A\right)=\text{Entropy }\left(C\right)-{\text{Entropy }}_{A}\left(C\right). \end{array}$$

The following are the unconditional direct values of class *C* attribute:

(2) $$\begin{array}{c} \text{Entropy }\left(C\right)=-\sum_{i=1}^{u}p_{i}{\text{log}}_{2}\frac{si}{n}. \end{array}$$

Assuming that attribute *A* has *V* value types, the conditional direct values of *C* can be calculated by dividing the dataset based on this:

(3) $$\begin{array}{c} {\text{Entropy}}_{A}\left(C\right)=-\sum_{j=1}^{v}\frac{s_{j}}{n}\left(-\sum_{i=1}^{u}\frac{s_{ij}}{s_{j}}\log\;2\frac{s_{ij}}{s_{j}}\right). \end{array}$$

Since describing attributes improves the categorization ability of attribute classes, the information gain value is positive, and the split information is introduced into the C4 algorithm to adjust the information gain. The following are the basic formulas for calculating attribute *A* split information values:

(4) $$\begin{array}{c} \text{SplitE}\left(A\right)=\sum_{j=1}^{v}\frac{s_{j}}{s}{\text{log}}^{2}\frac{s_{j}}{s}. \end{array}$$

Finally, the following information gain rates are obtained:

(5) $$\begin{array}{c} \text{GRatio}\left(S,A\right)=\frac{\text{Gain}\left(S,A\right)}{\text{SplitE}\left(A\right)}. \end{array}$$

In order to improve the uniformity and breadth of attribute division data, denominator with information gain rate can increase the number of attribute values, increase the amount of split information, decrease the rate of return, and also significantly remove the drawbacks of the number of attribute values.

### 3.3. Logistic Regression Algorithms

The basic theory of logistic regression algorithm is linear regression algorithm, which belongs to the classification algorithm. Its classification goal is to divide instances into any type of probability according to the value of self-confession energy. In this paper, *X*=(*X*_1_, *X*_2_, *X*_3_,…, *X*_*k*_) vector moisturizing data are used to describe the set of attributes, *Y* represents the attribute of data category, *P*(*X*) is the probability that *Y* occurs relative to *X*, and the following is the definition function:

(6) $$\begin{array}{c} P\left(X\right)=P\left(Y=1|X\right),\\ =\frac{1}{\left(1+e^{f\left(x\right)}\right)}. \end{array}$$

Nonlinear relationships among attributes are represented by *P*(*X*), and *f*(*X*) is a linear model based on linear regression theory, as follows:

(7) $$\begin{array}{c} f\left(x\right)=\beta_{0}+\beta_{1}x_{1}+\beta_{2}x_{2}+\cdots +\beta_{k}x_{k}. \end{array}$$

Logarithms of the above formulas are obtained:

(8) $$\begin{array}{c} f\left(x\right)=\text{In}\frac{p\left(x\right)}{1-p\left(x\right)}. \end{array}$$

The logistic regression model can reflect the impact of each *X* change on the classification prediction probability results, the sound value is the maximum solution on the logarithmic likelihood function of the predicted category attribute value vector, and the following is the logarithmic likelihood function expression:

(9) $$\begin{array}{c} \text{In}\left(L\left(\beta \right)\right)=\prod_{i=1}^{n}p{\left(x_{i}\right)}^{y_{i}}{\left[1-p\left(x_{i}\right)\right]}^{1-y_{i}}. \end{array}$$

### 3.4. Support Vector Machine Algorithms

A classification technique based on class distinctions is the support vector machine (SVM). For data instances with p unique properties, it may be seen as a p-dimensional vector. Choosing whether to divide the instances using a p-1-dimensional hyperplane is the transformation problem. With the help of this approach, we can separate two maximum edge hyperplanes. The support vector machine approach is best suited for problems involving binary classification. The dataset *D* is represented by the following formula, assuming that the *Y* class attributes have values between −1 and 1, where the attributes are given as *X* vectors in the P-1 dimension:

(10) $$\begin{array}{c} D=\left\{\left(x_{i},y_{i}\right)|x_{i}\in R^{P},y_{i}\in \left(-1,1\right),\;i=1,\ldots ,N\right\}. \end{array}$$

Within a data space composed of datasets, the decision boundary edge superplane is represented by the following formulas:

(11) $$\begin{array}{c} w\cdot x-b=\pm 1. \end{array}$$

Add the following constraints to allow data points to fall outside the edge line:

(12) $$\begin{array}{c} y\left(w\cdot x-b\right)\geq 1. \end{array}$$

So, the equivalent linear support vector machine maximizes the edge to minimize the objective function, which is calculated using the Lagrange multiplier formula:

(13) $$\begin{array}{c} f\left(w\right)=\frac{{\left\|w\right\|}^{2}}{2}. \end{array}$$

In order to soften the constraints for linear inseparable problems, the optimal segmentation plane can be obtained by adding a small *ξ*_*i*_ relaxation factor to all data instances in the above formula. By measuring the loss penalty factor *C* generated by the ignored outliers, the relaxation factor can be minimized. When dealing with the linear inseparable classification problem, the objective function should be adjusted as follows:

(14) $$\begin{array}{c} f\left(w\right)=\frac{{\left\|w\right\|}^{2}}{2}+C{\left(\sum_{i=1}^{N}\zeta_{i}\right)}^{k}. \end{array}$$

## 4. Cheerleading Referee Information Management System Based on Data Mining

Data mining is the process of examining and locating datasets. Data mining can identify the inherent patterns and connections in data as well as forecast future development trends using the data already available [14]. Data warehouses, relational databases, sophisticated database systems, and transaction databases may all benefit from data mining. Its generating process is efficient, clear, possibly beneficial, and effective. In general, data mining information reveals three qualities: efficacy, predictability, and practicability.

### 4.1. Information Management System Structure

Based on the data mining algorithm, this paper establishes the cheerleading referee information management system, in which the information management system (MIS) focuses on people, collects data by using software, computer hardware, office equipment and network communication, and realizes data transmission, storage, maintenance, and update, so as to comprehensively improve the operation efficiency and benefit of the information system and integrate the middle-level control. The high-level decision making and middle-level operation of enterprises have become a unified man-machine system [16].

One component corresponds to many frames when the management information system is separated into several different sections, and the mathematical index is utilized to forecast the structural quantity of the constituent system. Conceptual structure refers to the fundamental organization of management information systems. The MIS system is conceptually examined. Information processor, information source, information manager, and information consumer are some of its constituent parts. The major information comes from the information source. In order to give information managers and users, the information processor carries out the activities of information transmission, processing, and storage, converting the data into information or processed information. Managers are randomly selected as information users. Based on different information decision-making data on MIS, information managers analyze, design, develop, and coordinate different parts of the system, as shown in Figure 2.

### 4.2. Overall Structure of Cheerleading Referee Information Management System

This paper establishes a cheerleading referee information management system based on data mining. Its technical module components include background framework, front-end components, and database [17].  Figure 3 shows the basic sequence of system processing during user operation. The user submits the operation application on the system and uses the front-end data to verify and transmit the collected data. After verifying the data, complete the preprocessing based on the business logic, such as converting the digital format to generate statistical data, and complete the data assembly based on the business requirements. Multiple formats are defined in the database and background framework to realize the effective communication between the server and the client. When establishing information, the client program should send data to the server. After receiving the message sent by the client, the server will analyze the information and then further generate new data to return to the client.

The responsibility of the front-end component module is to realize the mutual communication between the customer and the system. The browser displays the operation page, and the user can complete various operations on the page. After that, the front-end component sends operation information to the background server to realize the mutual interaction with the background database. The most important part of react front-end is component, which can be split into multiple reusable and independent modules to develop front-end components. The background service, which receives the request and data information given by the foreground users, completes the preprocessing operation in accordance with the logical request established in advance and then sends the processed results back to the foreground, which is the logical centre of the system. The system calls the background to carry out the business after converting the JSON-type data given by the react foreground to Java Bean using the CXF framework. Data created on the system are saved and persistently stored using the database module. The system uses the Hibernate framework to do object relationship mapping and translates background service module execution into database operation to access database information.

### 4.3. System Main Structure Design

#### 4.3.1. System Functional Requirements

This paper comprehensively investigates the current situation of China's cheerleading referee information management system. At present, it can only deal with the openness of administrators, and the functional requirement data of the cheerleading referee system are shown in Table 1 [18].

According to the data shown in the above table, the functions of the cheerleading referee information management system are query function, new function, modification function, query referee information function, deletion function, import competition referee experience, import training experience, and exit.

#### 4.3.2. System Data Requirements

The information involved in evaluating the performance of cheerleading referees is shown in Table 2.

The items that account for a relatively low proportion of the information of cheerleading referees include “referee name,” “event name,” “team,” “event,” “effective frequency division rate,” “referee score,” and “effective frequency division number.” Since cheerleading is a subjective scoring item, the difference between the referee's evaluation score and the standard score is about 10 points, which are effective points. Therefore, after removing the highest and lowest scores given by the cheerleading referee, other scores are within the effective range. Further information about the referees involved in the training is shown in Table 3.

In the training information of cheerleading referees shown in Table 3, the lowest proportion is the training coach, only 64.6%, and the other information is higher than 90%.

#### 4.3.3. Designing the Main Structure of the System

Summarizing the above system requirements, the system is divided into six functional modules, namely, referee information, referee resume, query referee information, annual evaluation referee, event referee information, and training referee information.  Figure 4 shows the main structure of the front end of the system.

## 5. Analysis of Cheerleading Referee Information Management System

### 5.1. Analysis of the Number of Cheerleading Referees

This work develops the cheerleading referee information management system based on the data mining technique. Shaanxi Province is used as an example to examine the number of cheerleading referees when investigating the system's use [19]. It is helpful for Shaanxi Province to develop better strategies to enhance the refereeing ability and quality of cheerleading referees based on the analysis of the plants, the number of referees, and the evaluation data of cheerleading referees in the provincial and international competitions, as well as the comparison of refereeing data between first-class referees and higher-level referees and analysis of the issues.

According to each year, there are five types of experience and times of cheerleading referees going out to judge, namely, 0 times, 1–2 times, 3–5 times, 6–10 times, and more than 10 times [20]. The total number of people in this survey is 112.  Figure 5 shows the number of cheerleading referees each year. Only one person performs 0 times a year, accounting for 0.9% of the total, and 25 cheerleading referees perform 1 to 2 times a year, accounting for 22.3% of the total. The number of referees who perform three to five times a year is 33, accounting for 29.5% of the total. 23 cheerleading referees perform 6 to 10 times a year, accounting for 20.5%. There are 29 cheerleading referees who have performed more than 10 times, accounting for 25.9%. In this statistics, one person did not participate in the enforcement. According to statistics, cheerleading referees participate in the highest proportion of refereeing every year for 3 to 5 games.

Figure 6 shows the proportion of the number of first-class cheerleading referees and senior referees. According to the data in Figure 6, the proportion varies greatly with different levels of cheerleading referees. The number of senior referees participating in the competition is mostly 3–5 times a year. The number of referees performing more than 10 times a year accounts for 59.24% which is the highest proportion. The first-class referees have a large area, and the number of referees is mostly 1–2 times, 3–5 times, and 6–10 times. The number of referees more than 10 times accounts for 23.64%. This shows that senior referees have accumulated rich experience, so they perform more times.

### 5.2. Analysis of the Strength of Cheerleading Referees

When analyzing the application effect of cheerleading referee information management system, this paper judges according to the strength of cheerleading referee's on-the-spot judgment ability. The options set mainly include inaccurate grasp of the punishment scale, insufficient understanding of the new rules, lack of on-the-spot experience, audience interference, and others, as shown in Figure 7.

The failure to correctly comprehend the referee scale, according to the inquiry and analysis of the data of cheerleading referees in Shaanxi Province, was cited as the primary problem influencing accurate judgment during the on-the-spot execution by 45.6% of the referees. Each referee has unique characteristics, experiences, settings, educational backgrounds, and levels of rule comprehension and is directly influenced by their prior on-the-job refereeing knowledge. He is unable to fully comprehend the regulations and the circumstances on the cheering field during the on-the-spot referee, which leads to disagreements and interruptions in the competition process.

Among the referees, 38.83% pointed out that the lack of on-the-spot experience during on-the-spot execution was the main factor leading to wrong judgment. There are many factors causing the lack of on-the-spot experience, such as external factors, self-reasons, and so on. Referees are influenced by their personal work, and the short working hours of referees make them lack on-the-spot experience. 29.56% of the referees pointed out that the factor affecting the accuracy of on-the-spot judgment was the lack of in-depth understanding of the new rules. During the rapid development of cheerleading, the rules of cheerleading will be adjusted accordingly in order to meet the rapid development of cheerleading. Some cheerleading referees cannot effectively understand the adjusted rules, which makes it difficult to flexibly use the experience rules, while senior referees can fully understand the problem, and first-class referees do not fully understand the principle.

28.9% of the referees pointed out that the factor affecting the accurate judgment of temporary referees is the interference between athletes and coaches, and coaches and athletes will also directly interfere with the referees' refereeing effect. Therefore, referees should better deal with the relationship between cheerleading equipment and personnel and coordinate interpersonal relations, and referees must have very strong adaptability, good expression and communication ability, stable psychological quality, and self-control ability. With all those features, they can deal with the emergencies calmly. 17.9% of the referees pointed out that the audience can also affect the on-the-spot referee's ability, and the audience will also interfere with the referee's correct judgment during the cheerleading competition. Because the referee is not familiar with personal professional ability, he lacks strong psychological quality. 8.12% of the referees were influenced by other factors.

## 6. Conclusion

Cheerleading is a popular aerobics, which is deeply loved by people. It can not only exercise but also activate the atmosphere. It is an important international competition. An important role in the cheerleading competition is the cheerleading referee, which directly determines the fairness and impartiality of the cheerleading competition and has become a key part of people's attention. However, there is a common problem that the referee information cannot be effectively managed, which is still managed in the traditional paper way, resulting in management confusion. By investigating the demand analysis and system structure of cheerleading referees, the system structure is completed, and the cheerleading referee's information management system is established by using data mining algorithm. The analysis of cheerleading referees information system shows that most referees perform 3–5 times a year, and the percentage of referees who perform more than 10 times a year make up the biggest percentage which reach to 59.24%. The absence of on-the-spot experience, which accounts for 38.83% of the system's analysis of cheerleading referee strength, has the most impact.

## Figures and Tables

**Figure 1:** Data mining flowchart.

**Figure 2:** Information management system structure.

**Figure 3:** User operation sequence diagram.

**Figure 4:** System main structure.

**Figure 5:** Proportion of cheerleading referees.

**Figure 6:** Proportion of referees at different levels.

**Figure 7:** Analysis of the strength of cheerleading referees.

**Table 1:** System functional requirements.

Category	Frequency	Percentage
Add function	48	100
Query function	48	100
Modify function	48	96
Delete function	48	100
Referees retrieve information	48	100
Referees retrieve information	48	100
Import competition experience function	48	100
Exit function	48	100

**Table 2:** Cheerleading referee information.

Category	Frequency	Percentage
Event name	47	97.9
Referee's name	48	100
Participating team	48	100
Entries	42	87.5
Referee score	48	100
Effective frequency	35	72.9
Effective frequency division rate	34	70.8

**Table 3:** Cheerleading referee training information.

Category	Frequency	Percentage
Full name	48	100
Company	48	100
ID number	48	100
Level and score of cheerleading coach	46	95.8
Cheerleading referee report level and score	48	100
Skill referee report level and score	45	93.4
Training name	47	97.9
Training address	44	91.2
Train	31	64.6

## Data Availability

The datasets used and/or analyzed during the current study are available from the corresponding author on reasonable request.
